The article "Outcomes of Patients with Cervical Spinal Cord Injury Treated by Surgery and Their Prognostic Factors" was retracted in 2023. Reasons: signs of a paper mill; compromised peer review; unreliable results or conclusions.

# Outcomes of Patients with Cervical Spinal Cord Injury Treated by Surgery and Their Prognostic Factors

**DOI:** 10.1155/2022/8720290

**Published:** 2022-03-30

**Authors:** Xinfeng Wu, Qingpeng Song, Peihao Jin, Bo Liu

**Affiliations:** Department of Spine Surgery, Beijing Jishuitan Hospital, Beijing 100035, China

## Abstract

**Objective:**

To investigate the outcomes of patients with cervical spinal cord injury treated by surgery and their prognostic factors.

**Methods:**

We retrospectively analyzed 139 patients with cervical spinal cord injury treated by surgery at our hospital, who were admitted between January 2017 and December 2018. Depending on the Barthel index at last follow-up, the patients were divided into the recovery group (*n* = 60, Barthel index > 45) and the nonrecovery group (*n* = 79, Barthel index ≤ 45). General information of patients in the two groups was compared. The significant factors were further introduced into the logistic regression model. The poor prognostic factors of cervical spinal cord injury treated by surgery were analyzed, and specific nursing measures were taken.

**Results:**

There were significant differences in the duration of injury before admission, duration of injury before surgery, transportation and protection before admission, spinal canal invasion rate, and hormonal therapy within 8 h after injury between the patients achieving good postoperative recovery and those not (*P* < 0.05). Logistic regression analysis showed that all the factors above were prognostic factors for cervical spinal cord injury treated surgically.

**Conclusion:**

The duration of injury before admission, duration of injury before surgery, transportation and protection before admission, spinal canal invasion rate, and hormonal therapy within 8 h after injury were prognostic factors of patients with cervical spinal cord injury treated by surgery. The following factors should be considered for favorable outcomes: spinal protection during transportation to hospital, timely hormonal shock therapy to delay injury progression, and timely surgery to relieve pain. The spine is composed of cervical, thoracic, lumbar, sacral, and caudal vertebrae.

## 1. Introduction

The spine supports the trunk while walking upright, stooping, or bending. The spinal column encases the central nervous system, which governs limb movement [1, 2]. The cervical spinal segments are where the movement amplitude and frequency are higher. Fracture and dislocation of these segments are likely to induce structural or function injury of the cervical spine, which further causes spinal cord injury [3, 4]. Spinal fracture combined with spinal cord injury is a severe and complex traumatic disease. Falls from height and traffic accidents are the common causes of this disease, which presents with motor, sensory, sphincter, and autonomic nervous system disorders below the injury level. If not properly treated, spinal cord injury may lead to lifelong disability and secondary complications of other systems, which may be life-threatening [5, 6]. The best treatment for spinal fracture with spinal cord injury is surgical reduction of the fractured and dislocated spine plus spinal decompression. The purpose is to maintain spinal stability and protect and restore neurological functions. However, no consensus has been reached concerning the efficacy and prognostic factors of spinal fracture with spinal cord injury treated by the methods above [7, 8]. In this study, we enrolled 139 patients who were surgically treated for cervical spinal cord injury at our hospital from January 2017 to December 2018. The prognostic factors of the patients with cervical spinal cord injury treated by surgery were analyzed.

The article "Outcomes of Patients with Cervical Spinal Cord Injury Treated by Surgery and Their Prognostic Factors" was retracted in 2023. Reasons: signs of a paper mill; compromised peer review; unreliable results or conclusions.

## 2. Materials and Methods

### 2.1. General Information

We enrolled 139 patients who were surgically treated for cervical spinal cord injury at our hospital from January 2017 to December 2018. Inclusion criteria include (1) intact data without early withdrawal and (2) conforming to the diagnostic criteria developed by the American Spinal Injury Association (ASIA) [9]. Exclusion criteria include (1) severe infection, autoimmune diseases, or severe somatic diseases, (2) coagulation disorders, and (3) history of cervical spine surgery.

### 2.2. Methods and Observation Indicators

Data were collected from all patients. Depending on the Barthel index [10] at the last follow-up, the patients were divided into the recovery group (Barthel index > 45) and the nonrecovery group (Barthel index ≤ 45). The two groups of patients were compared in the following aspects: age, gender, course, cause of injury, transportation and protection before admission, spinal segment fractured, duration of injury before admission, duration of injury before surgery, spinal canal invasion rate, hormonal therapy within 8 h after injury, surgical approach, and preoperative traction. The prognostic factors were analyzed using the logistic regression model.

### 2.3. Statistical Analysis

All data were analyzed using SPSS 19.0 software. Counts were expressed as percentages and analyzed by the 03 test. Measurements were expressed as the mean ± SD and analyzed by the *t*-test. Binary logistic regression analysis was conducted. *P* < 0.05 indicated a significant difference.

## 3. Results

### 3.1. Poor Prognosis

Among the 139 patients (Frankel classification A 61 cases, B 7cases, C 31 cases, and D 40 cases) who were surgically treated for cervical spinal cord injury, 79 had a Barthel index ≤ 45, accounting for 56.83%.

The article "Outcomes of Patients with Cervical Spinal Cord Injury Treated by Surgery and Their Prognostic Factors" was retracted in 2023. Reasons: signs of a paper mill; compromised peer review; unreliable results or conclusions.

### 3.2. General Information

There were significant differences in the duration of injury before admission, duration of injury before surgery, transportation and protection before admission, spinal canal invasion rate, and hormonal therapy within 8 h after injury between patients achieving good postoperative recovery and those not (*P* < 0.05) (Table 1

### 3.3. Prognostic Factors

Logistic regression analysis identified duration of injury before admission, duration of injury before surgery, protection before admission, spinal canal invasion rate, and hormonal therapy within 8 h after injury as poor prognostic factors of patients with cervical spinal cord injury treated by surgery (Table 2).

## 4. Discussion

The incidence of spinal fracture with spinal cord injury has been rising yearly as traffic accidents are more common in modern society. Spinal fracture with spinal cord injury causes motor, sensory, sphincter, and autonomic nervous system disorders below the injury level. The patients' respiration, circulation, metabolism, and body temperature regulation are adversely influenced, and quality of life is severely affected [11, 12].

Cervical fracture and dislocation complicated by cervical spinal cord injury is a severe type of trauma, and the causes generally include traffic accidents, falls from height, and stumbling down, which may well cause death or disability [13]. At present, the best treatment for spinal fracture with spinal cord injury is surgical reduction of the fractured and dislocated spine plus spinal decompression, which can restore the normal alignment and stability of the damaged segment, relieve spinal cord compression, and create conditions for the recovery of nerve function [14, 15]. Although the surgical techniques for spinal fracture with spinal cord injury have matured, recovery of the patients after surgery is unsatisfactory [16]. In our study, among the 139 patients, 79 had a Barthel index ≤ 45, accounting for 56.83%. There were significant differences in the duration of injury before admission, duration of injury before surgery, transportation and protection before admission, spinal canal invasion rate, and hormonal therapy within 8 h after injury between patients achieving good postoperative recovery and those not (*P* < 0.05). Logistic regression analysis showed that all the factors above were prognostic factors of patients with cervical spinal cord injury treated by surgery. In light of the prognostic factors identified, we arrived at the following conclusions. (1) Duration of injury before admission: massive nerve cell death may occur within a few hours after cervical spinal cord injury. The longer the duration of injury before admission, the more delayed the standard treatment, such as dehydration therapy, hormone therapy, and neck immobilization. That is, the lower the chance of recovery after treatment. Therefore, the longer the duration of injury before admission, the worse the prognosis [17, 18]. (2) Duration of injury before surgery: it is generally believed that surgery should be performed within 72 h for patients with incomplete cervical cord injury. This is because severe nerve injury usually occurs after cervical spinal cord injury, presenting with apoptosis of gray and white matter cells within a few hours. Timely decompression can prevent and reduce secondary injury. The earlier the surgical decompression, the better the prognosis of patients with spinal cord injury [19–22]. (3) Transportation and protection before admission: the spinal cord without protection from the spinal column may be compressed and stretched if no proper protection is given during the transportation to the hospital. As a result, the spinal column and spinal cord injury may be aggravated. It is necessary to protect the spinal column at an early stage during the transportation process. When carried, the patients should have the head held with slight outward traction along the longitudinal axis of the body to align the head with the axis of the trunk. Moreover, swinging or torsion of the trunk should be avoided [23–25]. (4) Spinal canal invasion rate: the higher the spinal canal invasion rate, the more significant the decline of the conduction function of the spinal cord will be. As a result, the spinal cord is more greatly compressed. The spinal canal invasion rate is positively correlated with the degree of spinal cord compression. If the degree of spinal cord compression exceeds 50%, recovery may be almost impossible [26–28]. (5) Hormonal therapy within 8 h after injury: studies have shown [29–31] that high-dose methylprednisolone shock therapy within 8 h after injury shows moderate efficacy. If the patients are diagnosed and treated within 3 h after surgery, they can achieve better efficacy than if they are treated later (within 8 h). Worse prognosis of patients who were not treated by hormones within 8 h after injury was reported. In other words, high-dose methylprednisolone shock therapy within 8 h after injury improved prognosis. In addition, rehabilitation plays an important role. The SCI-FI [32] came up with measures of 5 subdomains of physical function: basic mobility, self-care, fine motor, wheelchair mobility, and ambulation in a conceptual structure that is unique to individuals with SCI. Kisala et al. and Tulsky et al. [33, 34] provide additional psychometric and interpretive information to support researchers and clinicians in their use of SCI-FI measures in research and practice.

The article "Outcomes of Patients with Cervical Spinal Cord Injury Treated by Surgery and Their Prognostic Factors" was retracted in 2023. Reasons: signs of a paper mill; compromised peer review; unreliable results or conclusions.

In conclusion, the duration of injury before admission, duration of injury before surgery, transportation and protection before admission, spinal canal invasion rate, and hormonal therapy within 8 h after injury were prognostic factors of patients with cervical spinal cord injury treated by surgery. The following factors should be considered to improve prognosis of the patients: strict strengthening during transportation to hospital, 8 hours in time hormonal shock therapy to delay injury progression, and 72 hours in time surgery to relieve pain.

## Figures and Tables

**Table 1:** General information in the two groups (*n* = 139).

General information		*n*	Nonrecovery group (*n* = 789)	Recovery group (*n* = 60)	*χ* ^2^	*P*
Age (years)	≤50	69	35	34	0.456	*P* > 0.05
	>50	70	44	26		
Gender	Male	122	70	52	0.013	*P* > 0.05
	Female	17	10	7		
Cause of injury	High energy	105	64	41	2.967	*P* > 0.05
	Low energy	34	15	19		
Transportation and protection before admission	Yes	108	55	53	6.891	*P* < 0.05
	No	31	24	7		
Segment fractured	C_3-5_	86	49	37	0.002	*P* > 0.05
	C_6_–T_1_	53	30	23		
Duration of injury before admission (h)	≤24	101	47	54	15.976	*P* < 0.05
	>24	38	32	6		
Duration of injury before surgery (h)	≤48	108	62	46	0.065	*P* > 0.05
	>48	31	17	14		
Spinal canal invasion rate (%)	>20	42	33	9	11.592	*P* < 0.05
	≤20	97	46	51		
Hormonal therapy within 8 h after injury	Yes	105	51	54	11.947	*P* < 0.05
	No	34	28	6		
Surgical approach	Anterior	78	44	34	0.344	*P* > 0.05
	Posterior approach	12	6	6		
	Anteroposterior approach	49	29	20		

**Table 2:** Prognostic factors of patients with cervical spinal cord injury treated by surgery.

Prognostic factors	*β*	S.E.	*f*	*P*	95% CI for EXP (*B*)	OR
Duration of injury before admission	0.511	0.097	1	0.001	1.7008 to 2.8374	1.796
Duration of injury before surgery	0.203	0.089	1	0.001	3.6926 to 4.1326	2.753
Transportation and protection before admission	0.229	0.068	1	0.001	2.7511 to 3.1911	2.647
Spinal canal invasion rate	0.232	0.039	1	0.001	1.4718 to 1.9118	1.529
Hormonal therapy within 8 h after injury	0.140	0.104	1	0.001	4.3418 to 4.7818	3.477

## Data Availability

The data used to support the findings of this study are available from the corresponding author upon request.
